RETRACTED

# Exosomes derived from human umbilical cord Wharton's jelly mesenchymal stem cells ameliorate experimental lymphedema

**DOI:** 10.1002/ctm2.384

**Published:** 2021-07-19

**Authors:** Zhao Ting, Yan Zhi‐xin, Tan You‐wen, Yang Fu‐ji, Sun Hui, Mao Fei, Zhu Wei, Xu Wen‐rong, Qian Hui, Yan Yong‐min

**Affiliations:** ^1^ School of Medicine Jiangsu University 301 Xuefu Road Zhenjiang China; ^2^ The Aflliated Changzhou No. 2 People's Hospital of Nanjing Medical University Changzhou China; ^3^ The Affiliated Hospital of Jiangsu University Jiangsu University Zhenjiang China; ^4^ The Affiliated Third Hospital of Zhenjiang Jiangsu University Zhenjiang China; ^5^ School of Medicine Jiangsu University 301 Xuefu Road Zhenjiang 212001 China

Dear Editor,

Acquired lymphedema is a complex disease caused by cancer treatment or parasitic infection and few effective treatments are available for lymphedema.^1^, ^2^, ^3^ It is urgently needed to develop new experimental approaches and therapeutic strategies.^3^ In this study, we address a new role and mechanism of MSC‐ex (human umbilical cord Wharton's jelly mesenchymal stem cells derived exosome) in lymphedema treatment. We found that MSC‐ex delivered Ang‐2 (angiopoietin‐2) promoted lymphangiogenesis by upregulating Prox1 (Prospero Homeobox 1) mediated Akt signaling. MSC‐ex can improve lymphatic function and ameliorate edema in a mouse model of acquired lymphedema.

MSC‐ex were isolated from the conditional medium of WJ‐MSC, which were negative for CD206 and positive for CD29, CD44 (Figure 1A,D). Exosomal markers CD9, CD63, CD81, and TSG101 were expressed in MSC‐ex, whereas Calnexin was not detected (Figure 1B,C). MSC‐ex showed a spheroid shape, and the size was about 130 nm (Figure 1E‐G). To investigate the effect of MSC‐ex on edema, we developed an acquired lymphedema model via surgical dissection of lymphatic vessels in the mouse tail (Figure 1H). As shown in Figure 1I, subcutaneously administered Dir labeled MSC‐ex localized in the injured tail at 24 h after treatment. MSC‐ex treatment promoted lymphatic drainage in lymphedema mice as injected methylene blue across the site of incision at week 6, which was not found in PBS treated mice (Figure 1J). The edema determined by tail diameter was persisted in mice treated by PBS. However, the edema was markedly reduced at week 2 in mice treated by MSC‐ex (Figure 1K). As lymphangiogenesis is crucial in lymphedema development after lymphatic ablation,^4^, ^5^ we analyzed the lymphatic anatomy and lymphangiogenesis in MSC‐ex treated animals. Relative to PBS‐treated animals, a relatively thinner dermis and epidermis was found in MSC‐ex treated mice (Figure 1L). Number of LYVE‐1^+^ (lymphatic endothelial hyluronan receptor‐1) lymphatics was also increased in MSC‐ex treatment group compared with those in PBS control (Figure 1M). These *in vivo* findings demonstrated that MSC‐ex can regenerate lymphatics and alleviate experimental lymphedema.

RETRACTED

**FIGURE 1:** MSC‐ex reduced lymphedema and enhanced lymphangiogenesis in vivo. (A) MSC markers of CD29, CD44, and CD206 detection by imaging flow cytometry. (B, C) Exosomal markers (CD9, CD63, CD81, TSG101) and non‐exosomal markers of Calnexin detection by imaging flow cytometry and western blot. (D) Representative images of MSC (20×). (E, F) Representative images of nano‐size vesicles photographed by transmission electron microscope (TEM) and atomic force microscope (AFM). Scale bar, 100 nm. (G) Nanoparticle tracking analyses of MSC‐ex in PBS. (H) Representative images of microsurgical ablation of major lymphatic conduits in the mouse (Hi). Schematic illustration of in vivo animal test for evaluating efficacy of MSC‐ex on lymphedema (Hii). (I) Distribution of Dir labeled MSC‐ex in mouse tail by in vivo fluorescent imaging 24 h post‐treatment. (J) Representative images of intradermal injection of methylene blue on day 42 resulted in transportation of the dye across incision site (n = 6). (K) Assessment of circumference directly at 0 cm, 1 cm, and 2 cm distal of incision site (n = 6; *P < 0.05 vs PBS, **P < 0.01 vs PBS). (L) Representative histology of mouse tail harvested on day 42. Dermal thickness was quantified (n = 6; **P < 0.01 vs PBS). Scale bar, 100 μm. (M) Representative images of immunohistochemical staining for LYVE‐1 positive lymphatics from mice treated with PBS, MSC or MSC‐ex on day 42. Number of LYVE‐1 positive lymphatics were quantified (n = 6; **P < .01 vs PBS). Scale bar, 100 μm. All data are presented as means ± SEM, Mann‐Whitney test. PBS, phosphate saline solution; MSCex, mesenchymal stem cells derived exosomes. LYVE‐1, lymphatic endothelial hyluronan receptor‐1

To determine whether MSC‐ex exert a direct effect on lymphangiogenesis, HDLEC (human dermal lymphatic endothelial cell) was incubated with PKH26 labeled MSC‐ex. Confocal imaging of immunofluorescence results showed that the labelled MSC‐ex mainly localized in the cytoplasm and around the nucleus at 12, 24, and 36 h after incubation (Figure 2A). MSC‐ex treatment dose‐dependently promotes tube formation, cell migration and proliferation of HDLEC (Figure 2B‐D). The level of LYVE‐1 was also enhanced time‐dependently following MSC‐ex treatment (Figure 2E‐F). We next studied the pathways that involved in MSC‐ex mediated lymphangiogenesis. Results showed that expression of the lymphangiogenic factors including Ang2, Prox1, p‐Akt was significantly increased with time in MSC‐ex treated HDLEC (Figure 2G).

RETRACTED

**FIGURE 2:** MSC‐ex exhibits dose‐dependent effect on lymphangiogenesis. (A) Representative fluorescent images of PKH26‐labeled MSC‐ex in HDLECs at 12, 24, and 36 h post MSC‐ex incubation. Scale bars, 10 μm. (B) CCK‐8 assay showing the effect of MSC‐ex on HDLEC proliferation at 24 h (n = 5; **P < .01 vs PBS). (C) Transwell migration assay of MSC‐ex treated HDLEC. (n = 5; **P < .01 vs PBS). Scale bars, 100 μm. (D) Matrigel tube formation of MSC‐ex treated HDLEC. (n = 4; *P < .05 vs PBS). Scale bars, 100 μm. (E) Representative immunofluorescent images of LYVE‐1 expression in PBS or MSC‐ex treated HDLECs at 24 h. Scale bars, 10 μm. (F) Western blot for LYVE‐1 in HDLEC treated with MSC‐ex at indicated time (n = 4; *P < .05 vs PBS). (G) Western blot for Ang2, Prox1, p‐Akt, and t‐Akt in MSC‐ex treated HDLEC at indicated time (n = 4; *P < .05 vs PBS). (H) Western blot for Ang1, Ang2, Prox1, and VEGFR3 in MSC‐ex or MSC from different batches. (I, J) Representative immunofluorescent images of Ang2 expression in HDLEC (n = 4; *P < .05 vs PBS, Scale bars, 10 μm.) and mouse tails (n = 4; *P < .05 vs PBS, Scale bars, 50 μm). All data are presented as means ± SEM, Mann‐Whitney test. HDLEC, human dermal lymphatic endothelial cells; MSC‐ex, mesenchymal stem cells derived exosomes; PBS, phosphate saline solution

We previously demonstrated that MSC‐ex contain functional proteins that can transfer to target cells for therapeutic tissue purpose.^6^, ^7^, ^8^ Then we sought to investigate the factors delivered by MSC‐ex role in lymphangiogenesis. We investigated the level of lymphangiogenic factors in MSC‐ex. Western blot analysis revealed that lymphangiogenic factors Ang2 but not Ang1, Prox1, VEGFR3 was detected in MSC‐ex and its derived MSC from different batches (Figure 2H). Immunofluorescence staining also confirmed that localization of human derived CD9 positive MSC‐ex both in HDLEC and in mouse tails lead to increased Ang2 expression in MSC‐ex treated mice but not in PBS control (Figure 2I and J). Taken together, MSC‐ex can promote *in vitro* lymphangiogenesis through its transfer of Ang‐2.

To confirm the role of Ang‐2 in MSC‐ex mediated lymphedema reduction, we analyzed the effect of MSC‐ex^Ang‐2^ (MSC‐ex with Ang‐2 overexpression) or MSC‐ex^shAng‐2^ (MSC‐ex with Ang‐2 knockdown) on lymphangiogenesis regulation. The level of Ang‐2 was increased in MSC‐ex^Ang‐2^ and decreased in MSC‐ex^shAng‐2^ respectively (Figure 3A). Consistently, cell proliferation, tube formation, and migration of HDLEC was enhanced in MSC‐ex^Ang‐2^ group (Figure 3B,C) and were interfered in MSC‐ex^shAng‐2^ group (Figure 3D and E). Furthermore, after injection into the mouse model of lymphedema, Ang‐2 expression in lymphatics was lower in MSC‐ex^shAng‐2^ group than which in MSC‐ex^shCtr^ group (Figure 3F). Evidence was also provided for the thickened dermis observed in MSC‐ex^shAng‐2^ treated mice, whereas MSC‐ex^shCtr^ treated animals showed a relatively thinner dermis in this model (Figure 3G). In addition, a significant reduction of the edema and restoration of lymphatic fluid drainage were found in MSC‐ex^shCtr^ group and Ang‐2 knockdown attenuated the reduction of MSC‐ex^shCtr^ on edema (Figure 3H,I). Thus, Ang‐2 knockdown delayed MSC‐ex mediated edema reduction, which was important in MSC‐ex promoted lymphangiogenesis.

RETRACTED

**FIGURE 3:** Prolymphangiogenesis effect of MSC‐ex on HDLEC was mediated by Ang2. (A) Western blot for Ang2 in MSC‐ex from MSC transfected with Lenti‐Ang2 (MSC‐exAng2) (Ai), Ang2‐shRNA (MSC‐exshAng2) (Aii) (n = 4; *P < .05 vs MSC‐exGFP). (B) Transwell migration assay (n = 5; *P < .01 vs MSC‐exGFP, Scale bars, 200 μm) and matrigel tube formation of MSC‐exGFP/MSC‐exAng2 treated HDLEC (n = 4; *P < .05 vs MSC‐exGFP, Scale bars, 100 μm). (C) CCK‐8 assay of MSC‐exGFP/MSC‐exAng2 treated HDLEC (n = 4; *P < .05 vs MSC‐exGFP). (D) Transwell migration assay (n = 4; *P < .05 vs MSC‐exshCtr, Scale bars, 200 μm) and matrigel tube formation of MSC‐exshCtr/MSC‐exshAng2 treated HDLEC (n = 4; *P < .05 vs MSC‐exshCtr, Scale bars, 100 μm). (E) CCK‐8 assay of MSC‐exshCtr/MSC‐exshAng2 treated HDLEC (n = 4; *P < .05 vs MSC‐exshCtr). (F) Representative immunofluorescent images of Ang2 expression in MSC‐exshCtr/MSC‐exshAng2 treated mouse tails. Relative mean fluorescence intensity (rMFI) was quatntied (n = 4; *P < .05 vs MSC‐exshCtr). Scale bars, 10 μm. (G) Representative histology of mouse tail harvested on day 28. Dermal thickness was quantified on day 28 in tail skin (n = 4; *P < .05 vs MSCexshCtr). Scale bar, 100 μm. (H) Representative images of intradermal injection of methylene blue on day 28 (n = 4). (I) Assessment of the circumference directly on day 28 after PBS, MSC‐exshCtr, and MSCexshAng2 treatment (n = 4; *P < 0.05 vs MSC‐exshCtr). All data are presented as means ± SEM, Mann‐Whitney test. PBS, phosphate saline solution; MSC‐ex, mesenchymal stem cells derived exosomes

Ang‐2 can regulate lymphatic differentiation, cellular junctions, and lymphatic sprouting and is crucial in lymphangiogenesis.^9^, ^10^ To corroborate the mechanism of MSC‐ex‐derived Ang‐2, the regulation effect of Ang‐2 on HDLEC lymphangiogenesis and Prox1/p‐Akt signaling pathway was studied. Overexpression of Ang‐2 significantly induced HDLEC migration, tube formation and proliferation (Figure 4A‐C,F), which were reversed by knockdown of Ang‐2 (Figure 4D,E,G). What's more, Prox1 and p‐Akt expression in HDLEC were upregulated by Ang‐2 overexpression (Figure 4H). Interestingly, overexpression of Prox1 in HDLEC increased p‐Akt expression (Figure 4I), whereas Prox1 knockdown resulted in decreased p‐Akt expression (Figure 4J). In addition, blocking p‐Akt with selective Akt inhibitor (MK‐2206) in HLDEC reversed Prox1 induced tube formation (Figure 4K,L). These data suggest that MSC‐ex transferred Ang‐2 increases lymphangiogenesis, at least in part, by modulating Prox1 mediated Akt signaling and Akt signaling is required for the HDLEC tube formation (Figure 4M).

RETRACTED

**FIGURE 4:** Ang‐2 enhanced HDLEC lymphangiogenesis by upregulating Prox1 mediated Akt signaling. (A) Western blot for Ang2 in HDLEC transfected with lenti‐GFP or lenti‐Ang2 (Ai), control shRNA (shCtr) or Ang2‐shRNA (shAng2) (Aii). (B, C) Transwell migration assay, matrigel tube formation of HDLEC transfected with lenti‐GFP or lenti‐Ang2. (n = 4; *P < .05 vs GFP, **P < .01 vs GFP). (D, E) Transwell migration assay, matrigel tube formation of HDLEC transfected with shCtr or shAng2. (n = 4; *P < .05 vs shCtr, ns, not significant). (F, G) Cell proliferation of HDLEC transfected with lenti‐GFP or lenti‐Ang2 (F), shCtr or shAng2 (G) by CCK8 assay. (n = 4; *P < .05 vs GFP, **P < .01 vs GFP). (H) Western blot for Prox1, p‐Akt, and t‐Akt in HDLEC transfected with lenti‐GFP or lenti‐Ang2 (n = 4; *P < .05 vs GFP). (I, J) Western blot for Prox1, p‐Akt in HDLEC transfected with lenti‐GFP, lenti‐Prox1, control shRNA (shCtr), Prox1‐shRNA (shProx1) (n = 4; *P < .05 vs GFP). (K) Western blot for p‐Akt in HDLEC transfected with lenti‐GFP, lenti‐Prox1, lenti‐Prox1/MK‐2206 (Akt inhibitor) treatment (n = 4; *P < .05 vs lenti‐Prox1). (L) Matrigel tube formation of HDLEC transfected with lenti‐GFP, lenti‐Prox1, lenti‐Prox1/MK‐2206 treatmen,t and quantification (*n* = 4; *P < .05 vs GFP, ^#^ *P* < .05 vs Prox1). Scale bars, 50 μm. All data are presented as means ± SEM, Mann‐Whitney test. (M) Schematic representation of hypothetic mechanism for Ang2‐enriched MSC‐ex mediating prolymphangiogenesis through upregulating Prox1 mediated Akt signaling

In summary, we presented a new evidence of MSC‐ex for experimental lymphedema reduction and revealed a mechanism of Ang‐2 regenerates lymphatics via Prox1/Akt pathway. Ang‐2 is an important factor for MSC‐ex mediated recovery from lymphedema. MSC‐ex may ameliorate experimental lymphedema through the delivery of Ang2. It is a promising therapeutic strategy to treat lymphedema.
